# Intelligent Analysis and Classification of Piano Music Gestures with Multimodal Recordings

**DOI:** 10.1155/2022/8232819

**Published:** 2022-06-13

**Authors:** Xunyun Chang, Liangqing Peng

**Affiliations:** Shaoyang University, Shaoyang, Hunan, China

## Abstract

In the traditional recording system, recording any music includes a sizeable instrumental setup and allocates space for the music players. Lighter and fewer devices are replacing larger instruments due to technological advancement and epidemic environmental conditions. This research focuses on text, but audio and video types are also considered. Multiple signal classification with a 5G-based wireless communication network algorithm is implemented to perform the automatic recording and classification of the music data. In this research, a multi-modal gesture recognition dataset is considered for analysis. The dataset was obtained using sensor networks and an intelligent system to record the musical gestures and classify the recorded gestures. The development of machine learning algorithms is not limited to similar technological concepts. Still, it extends to almost all other technical resources such as the 5G network, signal processing, networking, and all other technical resources. This would lead to additional engineering challenges that are utilized in most cases, such as the development of gestures with multi-mode recording. This research has proposed MSA with WCN algorithm to perform intelligent analysis and classification of piano music gestures and is compared with the existing *K*-Means algorithm and achieved an accuracy of 99.12%.

## 1. Introduction

Traditional piano instruction relies on professional piano trainers who pay attention to their students as they play the piano and point out their mistakes and defects. This approach frequently necessitates one-on-one tuition from a piano teacher [1]. As educational standards have risen, there is an increasing need for tools to analyze piano performances. As a result, there are fewer piano performance evaluation resources available. Computer technology can be used to evaluate and show a user's performance, allowing them to practise and improve their performance without the assistance of a piano teacher [2]. This system will benefit students and piano enthusiasts. Gestures have a significant role in the teaching and learning of musical instruments. They also aid in communication between educators and pupils [3]. Gesture-based communication is the sole way to gain the conceptual and communicative knowledge necessary to learn how to play a musical instrument, perform and interpret its musical material, and express its music [4]. If this is the case, and music-making is grounded in the educational system, it follows that gestures play a large part in music-making [5]. When observing someone's gait, for example, one might learn a lot about them, including their current emotional condition. This means that when it comes to gait analysis, people can think of a lot of different goals and levels of analysis [6]. For example, people can look at the goal of identifying the gait; people can also look at the goal of extracting the expressive content of the gait; information about the emotional state of the person; and people can look at the goal of describing the physical properties of the movement [7]. Many kinds of data must be digitised in order to analyze music's emotional influence. Some audio signals are broken down into their acoustic parts, like rhythm and timbre, and algorithms are used to find these parts and figure out how people feel [8]. Human emotions are not entirely taken into consideration by the music suggestion algorithm. A lot of people used traditional music playback methods that looked at things like the user's music library and playlists, rather than their own preferences [9]. Emotional distance is calculated by comparing the emotional features of several pieces of music, arranging them by emotional distance, and then categorising the attributes of each piece of music. While music performance suggestion systems have some limitations, individuals who usually listen to rock may struggle to find recommendations for hip-hop or R & B that evoke the same emotions [10]. A factor analysis of music aspects (popular and unpopular) is proposed in order to quantify the emotional processing of songs in music performances. Emotional traits in music would be given appropriate weights under this system. The literature examines Facebook posts and comments as well as human emotion data to better understand the algorithm employed in a music performance system to judge songs. Experiments have shown that by analyzing music emotions, the above music performance system can achieve an 80 percent preparation rate, improving the competitiveness of musical works [11]. For the purpose of addressing the issue of the musical performance system's expression of emotional content over the Internet, a study based on customization and network tagging is described in the literature [12]. It is necessary to use feature users in order to measure the degree to which an individual's personal propensity toward music feels similar to that of another. In order to develop a personalised recommendation based on commonalities, emotion acquisition, analysis, and aggregation are all used [13]. The researcher has investigated the impact of emotional factors on musical performance. Music may convey a wide range of human emotions, including joy, hope, and love [14]. Music's ability to convey a range of emotions is a difficult problem for intelligent recognition. As indicated, features (such as random tag set and multitag nearest neighbour) that retrieve human emotions from diverse musical expressions should be classified under music expressions to properly show this link, as described. For the issue of poor music performance label prediction, a method based on the music emotion vector space model has been developed in the literature [15]. Using a spatial model, SVM can categorise and recognise the emotions evoked by music performance systems. The results of this study have a significant correlation with the results of the vector space model-based method of identifying music's emotional content. It was developed by the researcher using the auditory model to develop the pitch-tracking approach that uses correlation graphs to generate the audio stream pitch spectra and then evaluate the pitch significance of each pitch. The shortest possible pitch interval is chosen once the pitch contenders have been quantified into music notes [16]. The development of robot dancing movements based on the construction of emotional shifts and music beat sequences was made possible using continuous emotional psychology and regression prediction models. Music's emotional content was linked to a model of acoustic features, and then they set up a regression to look at how the emotional content of music changes over time, says the researcher. Low-level acoustic elements like melodies and tones, as well as higher-level genres and styles, can be used to show how someone feels. They were reduced to a D-dimensional space, linked to semantic traits, and the *K*-nearest neighbour technique was employed [17]. The researcher requested the help of a group of 20 music experts to test the hypothesis that the rhythm and timbre of a piece of music can evoke positive or negative emotions like joy, sadness, fear, or tranquilly and also built a recommendation algorithm based on music sentiment after studying the emotions conveyed by cinema soundtracks. Two fuzzy classifiers were used to measure emotional intensity in order to determine the emotional content of music using a continuous emotional psychology model and a regression model. There are many ways to detect musical models using convolution neural networks, such as the researcher technique. The researchers used a two-way mismatch (TWM) pitch saliency computation to find vocal melodies [18]. This is because singing sounds have a lower attenuation rate than musical instrument sounds. Presented multi-modal deep learning makes use of a double convolution neural network. With the help of a depth model 370-Boltzmann machine, the relationship between audio and lyrics may be found [19]. The second section examines methods for categorising emotions in music performance systems, including the physical properties and processing of music signals. In the study's third section, eight different forms of emotional expression were discovered. There follows a discussion of the intelligent algorithm's SVM, KNN, and other models. This is the third time this method has been used to examine the emotional content of music [20]. Research shows that the proposed method is highly recognisable and requires little preparation.

## 2. Motivation of the Study

In the recent technological era, tremendous development in the information technology sector has caused all other sectors to collaborate to face a revolution and profit. Compared to traditional music recording processes, the current technology provides the best use of technology in the recording processes. Music and musical instruments are difficult to acquire in the traditional system if the musicians are in remote areas. Results corresponding to piano playing courses are analyzed in this study using the multi-modal gesture recognition dataset. This dataset contains virtually confirmed piano music gestures with multi-mode recording performances to notes labelled and audio waveforms. The multiple signal classification (MSC) algorithm with artificial intelligence (AI) support is incorporated into the dataset to analyze and classify the data. This MSC algorithm is used on wireless communication networks (WCN) and 5G network to classify transmitted signals after they have been recorded and updated. Normally, classifications are made with three distinct sections that fall under the components of accelerometer signal capturing with the assistance of a smartphone. Without the help of signals, we cannot move on in our lives, and in any case, there must be a link with the signals for every person in this world. Without the proper signal or network, it is impossible to contact a person or else to share information from one place to another. The majority of social media applications rely solely on these networks and signals to function. The machine learning algorithm that is being used here is operated on live signals, but here the author has briefly explained the labelled data validation, which helps by describing what kind of activity is being processed here.

## 3. Materials and Methods

While looking at ancient music playing mechanisms, music has been working as one of the symbols for inner peace since the 17th century. Most of the trending technology has been improved, and this would be the right time to update every individual according to the technological world. But here, the actual update is about artificial intelligence until only humans can understand the wordings and operate according to the other person's commands. Now, machines do interact with humans just by understanding human voices. Music has been made smaller in recent days, earlier to 20 years people used to watch movies only in theatres, and by rarity, people would have a television in their house. By the way, we have earbuds that have wireless connectivity in them right now. Biometrics are used to operate the systems, earbuds, laptops, etc. ElectroMyoGraphy (EMG) is used to analyze electron flow and muscle movement. EMG can be used to monitor the abnormalities behind the muscular organs [21]. Having some literature commands in-between the concept would make much interactive, likewise mean absolute value suits few of EMG data and also in finding out the muscle operations response. Electricity is being one of the mandatory things and there will not be anything possible without the purpose of electricity; in this competitive world, consumer's demand is the most important thing to be considered. As like similar to that the power signals do affect either transmission or the power distribution [22].

The multi-model dataset is considered in this study. This multi-modal is a combined information about the music dataset. This combined data will be of different file formats for the same piano music. Some of the default multi-modal formats include text, audio, and video and other types of files available in the dataset to continue the process of recording and classification of the recorded videos. These processes are depicted in Figure 1. The mode is supported with the intelligent server and monitoring device that are connected through wireless networking. In this figure, it can be seen that various modes of recordings are highlighted. The actual gesture recording of the piano music is given in the top left corner of the figure. In the process of recording, certain cameras and sensors are attached to the personal computer for the data transmission. ElectroEncephaloGraphic (EEG) is a device that is connected to the human brain to test the influence of music. EEG amplifiers are utilized for data acquisition and do a significant role of converting the electrical signals from the sensors to a digital format. This converted format is then stored to the database. Next, in the top right block represents the digital piano that can be used by the musicians during the remote recording of the music and to give real-time exposure to the movement of fingers during the play. Below the virtual piano is the musical notes that can be prepared and uploaded in the database. All the data collected can be stored to the database which is equipped with the intelligent system and connected with wireless networks. As the knowledge of machine learning requires a set of data and only after getting trained by the system user would get the actual output from the computer vision. In such case when the process is made with the help of wireless systems it means by there should be some signal generation in order to make avail of the data. To manage this power quality is being considered as one of the important things in the present scenario.

While the quality analysis would include similar things that are input signal, second thing is to preprocess the input signal to prepare it for the feature extraction and finally classifying the events in order to make proper analyzation. Apart from this, the main advantage of this intelligent database is to analyze the music and perform classification based on the genre, musician, music, duration of play, and so on.

### 3.1. Dataset

Multi-modal gesture recognition is considered in this research. This dataset contains gestures of various applications which includes finger and lip movements, facial expressions, body pose, and so on. Among those applications, piano music playing gesture is considered for the study. In order to supply the proper data collection to the system to make further prediction the way of passing the signals should be proper, for example, the signal processing methods would have various extraction tips which means the FFT, WPT, ST, HST, GT, etc., all the sets are combined in the process of optimized features. Dataset management is important to create a separate algorithm in order to create best recording but at the same time it is necessary to send it through a standardized network.

The structure of a smart piano music-playing recording system using wireless networking will analyze the piano music through realization technique. In addition, it offers a method to assess that the piano playing is trained with the piano instrument gestures with multi-mode records. Furthermore, this declaration simulates the musicians to provide updated music through the continuing playing and recording procedures.

Presume that there are *v* training tests (*G*_*n*_, *H*_*n*_)  as learning parameters for the wireless sensor network, where *G*_*n*_ is the device's eigenvalue and *H*_*n*_ is the expected data result. Assuming the aspect of the input signal is *t*, *G*_*n*_=(*x*_*n*1_, *x*_*n*2_,…, *x*_*nt*_) is used to demonstrate the support vectors of the *x* sample. *H*_*n*_=(*x*_*n*1_, *x*_*n*2_,…, *x*_*nt*_) is used to show the predicted output sequence of the *n* sample. And *R*_*n*_=(*R*_*n*1_, *R*_*n*2_,…,*R*_*nt*_)^*S*^ is used to identify the *n* sample's output variable measurement. If the density between the *i* neurotransmitter and the adjacent *j* neurotransmitter is *F*_*ij*_ then *F*_*ij*_=*F*_*ij*_, where *j* is the lower limit of the  *j* neuron.

Whenever a nicotinic receptor has been used as a real-valued unit *R*_*n*_=*R*_*n*_, the changes in the surface province *N*_*nj*_ of a *j* is neurotransmitter that can always be discussed as

(1) $$\begin{array}{c} N_{nj}=\sum_{i}F_{ji}R_{ni}-\sum \emptyset_{j}. \end{array}$$

Here, *R*_*ni*_ is the initial element's *i* neurotransmitter output, and the current element's *j* neurotransmitter output continues to follow, and  ∫(*N*_*nj*_) is a transfer function. The calculation of *R*_*ni*_ is given as

(2) $$\begin{array}{c} R_{ni}=\sum_{i=1}^{j=1}\left(N_{nj}\right). \end{array}$$

The development in these skill techniques can be used to train the system *R*_*ni*_ using a *G*_*n*_ which is a sigmoid transfer function. The main goal of the training courses is to calculate the learning algorithm (see (3))

(3) $$\begin{array}{c} G_{n}=\frac{1}{2}\sum_{j=1}^{s}{\left(l_{nj}-R_{ni}\right)}^{2},\\ Gj=\sum_{i=1}^{u}G_{n}. \end{array}$$

The following (4) is used in every training process ∇_*n*_ to reduce the time the *F*_*ji*_ error value depends on the differential

(4) $$\begin{array}{c} \varepsilon_{n}F_{ji}=\sum_{i=1}^{j}\mu \delta_{nj}R_{nj}. \end{array}$$

In (5), *ε*_*nj*_ describes the energy equipment

(5) $$\begin{array}{c} \varepsilon_{nj}=\sum_{j=1}^{n}\left(l_{nj}-R_{nj}\right)R_{nj}\left(1-R_{nj}\right). \end{array}$$

When *R*_*nj*_ represents its activation functions unit, the measurement will be performed as shown as

(6) $$\begin{array}{c} \mu_{nj}=R_{nj}\left(1-F_{nj}\right)\sum_{j}\mu_{nj}F_{ij}. \end{array}$$

Throughout the wireless sensor network, the instructing unit *h*_*nj*_, it is prudent to employ AI presented as mean and standard errors, as shown as

(7) $$\begin{array}{c} \text{AI}=\frac{1}{dv}\sum_{d=1}^{s}\sum_{j=1}^{s}{\left({\hat{g}}_{nj}-g_{nj}\right)}^{2}. \end{array}$$

In equations (8) and (9), *n* denotes the value that connects the *j*^*th* ^ hidden layer network to that same output unit weight vectors of a *β*_*j*_ node in the network and also the information nodes

(8) $$\begin{array}{c} R_{nj}=\sum_{j=1}^{n}\beta g{\left(x+k+t\right)}^{1/2}, \end{array}$$

(9) $$\begin{array}{c} g_{i}=\sum_{j=k+1}^{n}\beta_{j}\left(g+x+G_{j}+t_{c}\right). \end{array}$$

The rhythm sense is represented by *g* and *x* within the dataset. The music frequency time is specified by *t*_*c*_. The intelligent order is still on the lookout for a new region *G* within its visual range. If the region *G* could be revised any further within the visible region and the normal meets, *g*_1_ > *g*_2_ random behaviour could be evaluated using

(10) $$\begin{array}{c} G_{j}=\sum_{i=1}^{\text{random}}G_{i}+\text{rand }m\left(vis\right)-\text{ if}\left(g_{1}>g_{2}\right),\\ G_{\text{inex}}=\sum_{i=1}^{\text{random}}G_{i}+\text{random}\left(ste\right)*\left(G_{\text{max}}-G_{i}\right), \end{array}$$

random(*vis*) specifies as the visual range and random(*ste*) represents as the steps. It is comparable to the intensity of a piano music audio. It is a measure of a music signal's tonality and its spatial frequency components. It is calculated by utilizing

(11) $$\begin{array}{c} \text{Center}=\frac{\sum_{t=1}^{h}gF\left[g\right]}{\sum_{t=1}^{H}F\left[g\right]}. \end{array}$$

In the (11), *F*[*g*] is considered as the amplitude, and (12) is used to calculate the sequence-v spectral bandwidth.

(12) $$\begin{array}{c} \text{BW}={\left(\sum_{i}H\left(g\right){\left(\int \left(g\right)-f_{g}\right)}^{x}\right)}^{1/x}, \end{array}$$

where *H*(*g*) denotes the spatial magnitude.

The piano music gestures with multi-mode recording bandwidth below which a significant portion of spatial patterns energy, 95%, can be found. It is computed as in the following (13):

(13) $$\begin{array}{c} Fg=\frac{1}{2}\sum_{x}\text{sig}\left[n\left(o\right)\right]-\int \text{sig}\left[n\left(o-1\right)\right]g\left(g-o\right), \end{array}$$

(14) $$\begin{array}{c} \text{sig}\left[b_{t}\left(p\right)\right]=\sum \left\{\begin{array}{cc} 1, & H\left(g_{x}\right)\geq 0,\\ -1, & H\left(g_{t}\right)<0. \end{array}\right) \end{array}$$

The bearing is represented by *g*_*x*_, the paranoid time is represented by *H*_*x*_, the input variable just at specific frequency is represented by *b*_*t*_, and the outside situation at the original period is represented by *g*_*t*_. The information piano music transistor can be written as follows (14):

The relevance is signified by *g*_*x*_, the paranoid time is described by *H*_*x*_, the effective difference can be observed only at a specific frequency and is described by *H*_*t*_, and outside situation is described by *g*_*t*_. The piano music transformer information can be described as

(15) $$\begin{array}{c} H_{t}=\in \sum_{x=1}^{t}\left(H_{x}.\left[g.H_{t}\right]+G\right). \end{array}$$

The matrix associated with the input entrance is denoted by *g*, and the paranoid period is denoted by *H*_*i*_.

## 4. Results and Discussion

The data for this study was validated using the multiple signal classification (MSC) algorithm. The study's results were generated by this algorithm. Parameters such as music memory, standard score, and command and interpret have been used to better understand the use of WSN with AI in system analysis.

Table 1 represents recording of streamed online piano music gestures with multi-mode recording, there might be frequency delay. The signal for achieving high efficiency in online mode is supposed being a structure transformer for users within that developed framework. If a musician notices any contradictions in the audio, they can respond and review it for subsequent sections. According to the text, AI will support in choosing different musicians and having to play audio/video through the wireless sensor network. Its methods within dataset will be updated by AI. According to the signals and machine learning concept, there are different classifiers, whereas the first important thing is the neural networking concept, second is to manage the genetic algorithm, third process is to manage the fuzzy logic to manage the miscellaneous process, and finally creating a support vector to process all classifiers. Before understanding about the error system, it is important to analyze the signals and computers that learn, there are separate software in order to match the audio signals with the video formats, if this could be made automatically by the systems then the work might be easier to complete and at the same time the user would get enough accuracy from it. Moreover, the machine learning concepts are introduced to get enough accuracy from the system at the same time there should not be any time delay to complete the process.

Figure 2 depicts the frequency analysis used in audio/video, text, and image. It is possible to extrapolate from this figure. The role of the controller is played by the musician who is in charge of the recording of the corresponding music. After the resources have been designed, they will be forwarded to the operations department, which will play the video based on the user's request. The quality of the video will be analyzed in the testing facility, and the duration and musician's information will be updated. Whether there is an issue, a monitor alarm will be engendered and conveyed to the executive and command office for further resource updates. The classification of piano music gestures with multimode recording (image, audio/video, image) with respect to testing (85%), training (84%), and frequency (92%) analysis for online piano classes (refer Figure 2).

The structure of such a smart piano music-playing recording process based on wireless networking will be used to analyze the realization technique of the piano recorded music process. Furthermore, it provides a method for assessing piano playing that is trained with piano playing gestures through multi-modal formats that are stored in the database. Musical recording is a method of sharing data which does involve information exchange. As Table 2 demonstrates the training and testing frequency analysis for the data Format image, audio/video, text for training and testing frequency the mean (91.33%), standard deviation (92.76%) and size (GB) training and testing frequency (65.46%) piano music gestures with multi-mode.

The Declarative language is a type with a modelling process and the ability to consider intelligently. It is related to the field of graphics but also information system's comprehension, and it includes propositions and judgment comprehension cases. The Declarative programming term is commonly used in datasets, ordinary, mathematical results, completely credible, insufficient credibility, automatic recognizing, and in other fields. As shown in Figure 3 it is not only widely used in music recording and the quantifier but also in mathematical expression framework of piano music gestures with multi-mode performance.

Table 3 illustrates the human work analysis as organizers of the International Piano-e-Competition to create the raw data shown in this dataset. The representation found in each competition installment, which is concert-reliable and credible pianos with an enhanced recording of multimodal gesture recognition capture and recording system has been addressed. The level of detail of the confirmed multi-modal gesture recognition data is high enough so the competition's opening act stage (refer to Table 3) can be evaluated remotely by having listened to contestant productions reproduced out over wire on that other Declarative instruments. Where combining the process of signal matching with the help of machine learning module, it is kind of two-step verification process whereas according to the field signal procession would manage with the audio signals. When this process is done by a system there are some alternatives in the procedures, for example analyzing the error report will be much easier in accordance with the computer vision. And here the network does not matters much.

The various piano music evaluations of such an audio signal are composed of piano music gestures with multi-mode able to transmit communication signal characteristics (Table 4). They are not only qualitatively motivated but also classify the distinctness of a rhythm sense signal in the sequential or frequency field. Because music varies (audio/video, image, text) so much (see Figure 4), physiological feature extraction and interrelated musical frames are important.

Even though music varies so much (see Figure 5), physiological feature extraction is done in short intersecting skylights. The analysis in the above figure is based on the number of users who reviewed the digital piano music learning classes concerning the frequency of the music. In some cases, the frequency and rhythm sensations appear to have inverted values about the user's response.

An audio wave signal's parameters are made up of various aspects of a piano music signal. They are not conceptually motivated, nor do they classify the distinctness of a piano signal in the space-time or frequency field (refer to Table 5). In the considered music composed by the piano musician, there are minor differences in time, frequency, and rhythm sensation.

Music recordings can be conducted through online using artificial intelligence in wireless networks. Artificial intelligence is used in application to help with the automatic playback of recorded videos. An Immc1 also plays an important role in suggesting tracks for users based on their needs and the comments they leave. The AI technique will update the database with all of the users' communication and responses. The music signal classification concept is implemented as an artificial intelligence technique to classify newly updated music information and update in the corresponding type of music. The steps for calculating the score for the online piano class are as follows: Both of these performances are represented by reduced lettered components. In Figure 6 Node (1) music performance results from equivalent to similar, Node (2) removes the most similar performances to leave an interference floor, and Nodes (3) and (4) insert additional comparable performance related appearances one at a time to see how well they can obstruct the noise surface. Specifically, the model's performance for musical instrument recognition is improved in addition to designing the model on the basis of a neural network and optimizing the structure. The test results reveal that an AI-based instrument recognizing model can meet the requirements of piano music gestures with multi-mode recording and hence increases the user's involvement in gaining knowledge about piano music gestures with multi-mode recording learning. Even the computers do analyze the accuracy in terms of matching the features but machine learning has an important role to match the further featuring at every single step process.

Brain waves outperform sound waves as an update to a machine learning model because they can be used to analyse the system's own sound waves. For example, just by using a few sensors, the machine is trained to analyze the human brain waves and asked to do the particular task as the waves function in the brain. Here the entire process proves the importance of signals and how the signals are processed in the form of utilizing the specific patterns. Noise is always being considered as the disturbance, in such cases, the sensors are modified to remove the noise from the brain waves. And the final thing is to prepare a package that stores the necessary information that is to be collected from the human brain. Even though the procession does not care more if the computer vision completes its work in a better way than the upcoming works do relate with the algorithm that is designed in accordance with the matched machine learning. Here the (refer Table 6) process of understanding the concepts is being further distinguished by the system and it makes predictions to understand whether the users tell them to move their hands or else he used to have their hands in a rest position. This kind of system with proper network usage can be used for people with limited mobility to control certain devices just by using their brain waves.

## 5. Conclusion

Traditionally, while recording any kind of music, a big instrumental setup is required and room is set aside to accommodate all of the musicians. As technology advances and environmental circumstances worsen, heavier and more numerous instruments are being phased out in favour of smaller, lighter ones. The automatic recording and classification of music data are accomplished through the use of a wireless communication network algorithm known as multiple signal classification. 5G networks and an intelligent system were used to record musical gestures and identify the recorded gestures to produce the dataset. The proposed model has obtained an accuracy of 99.12%. For training, video analysis has been recorded for this study. For future study, it is highly recommended to consider pre-recorded and live recorded videos.

## Figures and Tables

**Figure 1:** Model of the proposed piano music recording.

**Figure 2:** Classification of dataset in piano music gestures with multi-mode recording for testing frequency analysis using MSA with WCN algorithm.

**Figure 3:** The MSA with WCN algorithm with artificial intelligence using analysis of frequency in the effective use of piano music gestures with multi-mode (image, audio/video, image).

**Figure 4:** Performance analysis of piano music based on rhythm sense and communication command using MSC with WCN algorithm.

**Figure 5:** The recording system's effect in the evaluation of piano music gestures.

**Figure 6:** Performance analysis of piano music classification using artificial intelligence in wireless sensor networks.

**Table 1:** Analysis of dataset using MSC with WCN algorithm.

Dataset parameter	MSC with WCN algorithm	Structure converter	Dataset
Audio/video	163	243	547
Image	187	262	542
Text	195	246	678

**Table 2:** Testing and training frequency analysis result for piano music gestures with multi-mode (image, audio/video and image).

Process	Data format	Mean	Standard deviation	Size (GB)
Testing	Image	1.54	275	65.87
	Video/Audio	2.89	365	72.64
	Text	1.65	245	64.23

Training	Image	1.67	162	39.46
	Video/Audio	1.89	203	42.12
	Text	1.23	153	32.46

Frequency	Image	1.14	242	48.69
	Video/Audio	2.12	239	47.23
	Text	1.89	212	34.12

**Table 3:** The human work analysis for the piano music gestures with multi-mode (image, audio/video, image) using MSA with WCN algorithm.

Human works	Audio/video	Image	Test	Accuracy (%)
Objective	1544	374	126	92
Expert with extensive experience	1417	342	138	94
Dataset	1505	332	153	96
Ordinary dependable	2418	335	176	95
Insufficient credibility	2634	527	158	93
Completely credible	1757	368	165	97

**Table 4:** Performance analysis result piano music based on rhythm sense and communication command using MSC with WCN algorithm.

Piano musician		Audio/video	Image	Text
Piano music 1	Overall evaluation	0.983	0.765	0.812
	Communication command			
	Rhythm sense			

Piano music 2	Overall evaluation	0.8783	0.887	0.834
	Communication command			
	Rhythm sense			

Piano music 3	Overall evaluation	0.989	0.834	0.865
	Communication command			
	Rhythm sense			

Piano music 4	Overall evaluation	0.981	0.993	0.983
	Communication command			
	Rhythm sense			

Piano music 5	Overall evaluation	0.956	0.858	0.892
	Communication command			
	Rhythm sense			

Piano music 6	Overall evaluation	0.978	0.887	0.795
	Communication command			
	Rhythm sense			

Piano music 7	Overall evaluation	0.892	0.892	0.787
	Communication command			
	Rhythm sense			

Piano music 8	Overall evaluation	0.834	0.781	0.895
	Communication command			
	Rhythm sense			

Piano music 9	Overall evaluation	0.745	0.856	0.998
	Communication command			
	Rhythm sense			

Piano music 10	Overall evaluation	0.967	0.971	0.893
	Communication command			
	Rhythm sense			

**Table 5:** Frequency analysis in piano music gestures with multi-mode recording.

Piano music		Time (s)	Frequency	Rhythm sensation
Music 1	Audio/Video	0.754	0.764	0.814
	Image			
	Text			

Music 2	Audio/Video	0.816	0.677	0.846
	Image			
	Text			

Music 3	Audio/Video	0.882	0.754	0.717
	Image			
	Text			

Music 4	Audio/Video	0.866	0.827	0.663
	Image			
	Text			

Music 5	Audio/Video	0.793	0.774	0.788
	Image			
	Text			

Music 6	Audio/Video	0.767	0.795	0.735
	Image			
	Text			

Music 7	Audio/Video	0.844	0.717	0.778
	Image			
	Text			

Music 8	Audio/Video	0.826	0.862	0.764
	Image			
	Text			

Music 9	Audio/Video	0.825	0.748	0.897
	Image			
	Text			

Music 10	Audio/Video	0.823	0.599	0.691
	Image			
	Text			

**Table 6:** Comparison result analysis of piano music classification using artificial intelligence in wireless sensor networks.

Algorithm	Time (s)	Frequency	Rhythm sensation	Overall accuracy (%)
MSA with WCN algorithm	0.754	0.764	0.814	99.12

Existing method: K-means	0.816	0.677	0.846	94.35

## Data Availability

The data used to support the ﬁndings of this study are available from the corresponding author upon request.

## References

[1] Lee S. J., Seo B. G., Park D. H. (2018). Development of music recommendation system based on customer sentiment analysis. *Journal of Intelligence and Information Systems*.

[2] Khoeurn S., Yun S. K. (2017). Sentiment analysis engine for Canadian music industry re-building. *Journal of the Korea Society for Simulation*.

[3] Gómez L. M., CáCeres M. N. Applying data mining for sentiment analysis in music.

[4] Jing L. I., Lin H., Ruimin L. I. (2012). Sentiment vector space model based music emotion tag prediction. *Journal of Chinese Information Processing*.

[5] Chen C., Li Q. (2020). A multimodal music emotion classification method based on multifeature combined network classifier. *Mathematical Problems in Engineering*.

[6] Huang M., Rong W., Arjannikov T., Jiang N., Xiong Z. Bi-modal deep Boltzmann machine based musical emotion classification.

[7] Schiavio A., Høffding S. (2015). Playing together without communicating? a pre-reflective and enactive account of joint musical performance. *Musicae Scientiae*.

[8] Chang A., Livingstone S. R., Bosnyak D. J., Trainor L. J. (2017). Body sway reflects leadership in joint music performance. *Proceedings of the National Academy of Sciences*.

[9] Ambroise Grandjean G., Hossu G., Bertholdt C., Noble P., Morel O., Grangé G. (2018). Artificial intelligence assistance for fetal head biometry: assessment of automated measurement software. *Diagnostic and Interventional Imaging*.

[10] Zhang P., Xu X., Qin X. (2020). Evolution toward artificial intelligence of things under 6G ubiquitous-X. *Journal of Harbin Institute of Technology*.

[11] Pitt C. S., Bal A. S., Plangger K. (2020). New approaches to psychographic consumer segmentation. *European Journal of Marketing*.

[12] Hsieh Y.-Z., Lin S.-S. (2020). Robotic arm assistance system based on simple stereo matching and Q-learning optimization. *IEEE Sensors Journal*.

[13] Bousquet-Jette C., Achiche S., Beaini D., Law-Kam Cio Y. S., Leblond-Ménard C., Raison M. (2017). Fast scene analysis using vision and artificial intelligence for object prehension by an assistive robot. *Engineering Applications of Artificial Intelligence*.

[14] Heer J. (2019). Agency plus automation: designing artificial intelligence into interactive systems. *Proceedings of the National Academy of Sciences*.

[15] Mutsuhiro N. (2018). Utilization of biofeedback in an age of information and communication technology and artificial intelligence: industry-academia-government cooperation. *Japanese Journal of Biofeedback Research*.

[16] Caramiaux B., Tanaka A. Machine learning of musical gestures: principles and review.

[17] Donnarumma M. (2015). Biophysical music sound and video anthology. *Computer Music Journal*.

[18] Fiebrink R., Caramiaux B. (2018). The machine learning algorithm as creative musical tool. *The Oxford Handbook of Algorithmic Music*.

[19] Li H. (2020). Piano automatic computer composition by deep learning and blockchain technology. *IEEE Access*.

[20] Shuo C., Xiao C. (2019). The construction of internet + piano intelligent network teaching system model. *Journal of Intelligent and Fuzzy Systems*.

[21] Kumagai Y., Matsui R., Tanaka T. (2018). Music familiarity affects EEG entrainment when little attention is paid. *Frontiers in Human Neuroscience*.

[22] Kumagai Y., Arvaneh M., Tanaka T. (2017). Familiarity affects entrainment of EEG in music listening. *Frontiers in Human Neuroscience*.

